# Human Microbe-Disease Association Prediction by a Novel Double-Ended Random Walk with Restart

**DOI:** 10.1155/2020/3978702

**Published:** 2020-08-10

**Authors:** Di Wang, Yan Cui, Yuxuan Cao, Yuehan He, Hui Chen

**Affiliations:** ^1^Department of Nuclear Medicine, Harbin Medical University Cancer Hospital, Harbin, China; ^2^Department of Urology, Harbin Medical University Cancer Hospital, Harbin, China; ^3^Harbin Medical University College of Bioinformatics Science and Technology, Harbin, China

## Abstract

Microorganisms in the human body play a vital role in metabolism, immune defense, nutrient absorption, cancer control, and prevention of pathogen colonization. More and more biological and clinical studies have shown that the imbalance of microbial communities is closely related to the occurrence and development of various complex human diseases. Finding potential microbial-disease associations is critical for understanding the pathology of a few diseases and thus further improving disease diagnosis and prognosis. In this study, we proposed a novel computational model to predict disease-associated microbes. Specifically, we first constructed a heterogeneous interconnection network based on known microbe-disease associations deposited in a few databases, the similarity between diseases, and the similarity between microorganisms. We then predicted novel microbe-disease associations by a new method called the double-ended restart random walk model (DRWHMDA) implemented on the interconnection network. In addition, we performed case studies of colon cancer and asthma for further evaluation. The results indicate that 10 and 9 of the top 10 microorganisms predicted to be associated with colorectal cancer and asthma were validated by relevant literatures, respectively. Our method is expected to be effective in identifying disease-related microorganisms and will help to reveal the relationship between microorganisms and complex human diseases.

## 1. Introduction

Microorganisms include bacteria, archaea, protozoa, fungi, and viruses. There are different types of microorganisms on the human body and in the cavity connected to the outside world, such as the oral cavity, respiratory tract, intestinal tract, and urogenital tract [1, 2]. Microbes play important roles in human health, metabolism, immune defense, nutrient absorption, cancer control, and prevention of colonization of pathogens [3]. Microorganisms of the human body are mainly distributed on the body surface, intestine, and oral cavity, and the types and numbers of microorganisms are different. Among them, the number of microorganisms in the intestine is about ten times that of the body's own cells. In nature, the density of microorganisms isolated from the colon is the highest, and 60% of the dry weight of human feces is bacteria [4].

Numerous studies have shown that many diseases are related to changes in microorganisms. For example, patients with type 2 diabetes have been found to have moderate intestinal microecological disorders and lack of butyric acid-producing bacteria [5]. Intestinal microbial diseases lead to intestinal immune system dysfunction. For patients with irritable bowel syndrome (IBS), the number of chronic inflammatory cells in the colonic mucosa of increases, a large number of T cells are activated, and the expression of inflammatory reactions is accelerated [6]. In addition, epidemiological studies have shown that common mental illnesses such as autism and schizophrenia are associated with perinatal pathogen infections [7–11].

As mentioned above, discovering the potential links between microbes and diseases allows us to better understand the mechanisms by which disease is formed and developed. By regulating the microbial environment, medical solutions for disease prevention, diagnosis, treatment, and prognosis can be provided to some extent. In previous biological or clinical experimental research methods, it took a lot of time and cost to obtain a new connection between microorganisms and disease. In recent years, many computational biology methods have provided new and effective tools for identifying the key links between microorganisms and disease. Ma et al. constructed a microbe-disease association data pants called HMDAD, which can help study the relationship between microbes and diseases [12], and provide data support for various calculation methods to predict new associations

In recent years, machine learning algorithms have achieved good performance in various fields [13]. At present, various machine learning algorithms have been used in the prediction of the association between microorganisms and diseases and have achieved good performance. As such, Chen et al. established a microorganism-human disease association network and further developed a new KATZ metric calculation model for the prediction of human microorganism-disease association (KATZHMDA) under the premise that similar-function microorganisms tend to the following assumptions [14]. Huang et al. [15] proposed a path-based human microorganism-disease association prediction (PBHMDA) method that integrates the identified nuclear-similarities of disease-microbe relationships and Gaussian interaction spectra into a heterogeneous network of diseases and microorganisms. The model traverses all possible pathways between microbes and diseases. A novel depth-first search algorithm is used to predict the microorganisms most likely to be associated with the disease. In addition, Wang et al. [16] proposed a new computational model of Laplace regularized least squares to reveal potential disease-related microorganisms. LRLSHMDA applies a semisupervised learning framework. In this model, a microbial similarity network and a disease similarity network are constructed based on the Gaussian interaction spectrum kernel similarity calculated from known disease-disease associations, and the cost function in the microbial space and disease space is then constructed and optimized integrating the optimal classifier function to calculate the correlation probability of microbial disease pairs. Although the reliable prediction performance of LRLSHMDA has been verified, the model still has some shortcomings and needs further improvement. For example, the number of proven microbial associations is too small, and a sparse network of known associations may affect the predictive performance of the model. Shen et al. [17] combined the known similarity of microbe-disease association with the nuclear similarity of the Gaussian interaction spectrum; a collaborative matrix decomposition calculation model was established for the microbial-disease association prediction (CMFHMDA) of humans and diseases. A special matrix decomposition algorithm is proposed to update the correlation matrix between microorganisms and diseases and infers the microorganisms most likely to be related to diseases. However, the performance of this model needs improvement.

In summary, though the tremendous progress made in computing predictions of microbial-disease associations, there are still some limitations. In order to better reveal the association between microbial diseases, based on the known heterogeneous network consisting of microbial-disease association and Gaussian interaction contour kernel similarity, we propose a computational model based on a double-ended restart random walk to predict disease-related microorganisms. To prove the superiority of the DRWHMDA algorithm, we applied the 5-fold CV and global LOOCV to evaluate the prediction performance of DRWHMDA. In addition, we used DRWHMDA for case studies of two diseases.

## 2. Materials and Methods

### 2.1. Materials

The general workflow of DRWHMDA is shown in Figure 1. First, we need to preprocess the data. The original data comes from a microbe-disease association dataset named HMDAD constructed by Ma et al. [13]. HMDAD contains 483 artificially planned microbiological associations involving 39 diseases and 292 microorganisms. Because there are multiple evidences for some associations, we extracted 450 different disease-microbial associations. Secondly, based on these known microbial-disease associations, we constructed disease networks, microbial networks, and microbial-disease related networks, respectively. Here, *N*_*d*_ = 39 indicates the number of diseases, and *N*_*m*_ = 292 indicates the number of microorganisms. Finally, a two-terminal random walk is performed through a heterogeneous network. Combine different prediction scores into the final associated prediction probability according to the linear combination.

### 2.2. Symptom-Based Disease Similarity (SDM)

In the field of information retrieval, text documents or concepts are usually represented by feature vectors. Here, we describe the vector *d*_*j*_ of each disease *j* through symptoms.

(1) $$\begin{array}{c} d_{j}=\left(w_{1,j},w_{2,j},\cdots ,w_{n,j}\right), \end{array}$$

where *w*_*i*,*j*_ quantifies the strength of the association between symptom *i* and disease *j*. The prevalence of different symptoms and diseases is very different. In order to solve this heterogeneity, we do not use absolute co-occurrence *w*_*i*,*j*_ to measure the strength of the association between symptom *i* and disease *j*, but the term frequency and the reciprocal of the document frequency *w*_*i*,*j*_.

(2) $$\begin{array}{c} w_{i,j}=w_{i,j}\log\frac{N}{n_{i}}, \end{array}$$

where *N* represents the number of all diseases in the data set and *n*_*i*_ represents the number of diseases with symptom *i*.

Therefore, the similarity between the vectors *d*_*x*_ and *d*_*y*_ of the two diseases *x* and *y* is calculated as follows:

(3) $$\begin{array}{c} \cos\left(d_{x},d_{y}\right)=\frac{\sum_{i}d_{x,i},d_{y,i}}{\sqrt{\sum_{i}{d_{x,i}}^{2}}\sqrt{\sum_{i}{d_{y,i}}^{2}}}. \end{array}$$

The cosine similarity ranges from 0 (no shared symptoms) to 1 (identical symptoms).

### 2.3. Effect of Gaussian Interaction Spectroscopy Nuclear Similarity on Disease

Based on the assumption that diseases with similar phenotypes always share similar associations and nonassociative patterns with functionally similar microorganisms, the Gaussian interaction distribution kernel similarity between disease and disease can be further calculated. We define the binary vector VP(*d*_*i*_) to represent the interaction curve of disease *d*_*i*_, which can be obtained by observing whether *d*_*i*_ is known to be associated with each microorganism (i.e., the *i*th row of the adjacency matrix). Then, after calculating the similarity value between disease pairs, the Gaussian interaction distribution kernel similarity matrix (KD) can be constructed.

(4) $$\begin{array}{c} \text{KD}\left(d_{i},d_{j}\right)=\exp\left(-\gamma_{d}{\left|\left|\text{VP}\left(d_{i}\right)-VP\left(d_{j}\right)\right|\right|}^{2}\right) \end{array}$$

(5) $$\begin{array}{c} \gamma_{d}=\gamma \prime_{d}/\left(\frac{1}{nd}\overset{nd}{\underset{i=1}{\sum }}{\left|\left|\text{VP}\left(d_{i}\right)\right|\right|}^{2}\right) \end{array}$$

The parameter value *γ*_*d*_ controls the bandwidth of the Gaussian kernel. As shown in (5), *γ*′_*d*_ can be further calculated by dividing the new bandwidth parameter *γ*′_*d*_. The average of each disease is associated with microorganisms. Here, we *γ*′_*d*_ = 1 according to previous research [18].

From the above, we can see that the similarity of the Gaussian interaction spectrum kernel is only based on adjacency matrix *A*. If we want to effectively and scientifically predict potential disease-related microorganisms, it is necessary to incorporate other data sets similar to the Gaussian interaction spectrum kernel, recorded in PubMed bibliography based on disease and corresponding symptoms. Zhou et al. (2014) calculated similarities between diseases and established a symptom-based human disease network (HSDN). Here, we synthesize the Gaussian interaction spectrum kernel similarity of disease KD and symptom-based disease similarity SDM to obtain symptom-based disease similarity SD, and SD is calculated as follows:

(6) $$\begin{array}{c} \text{SD}=\frac{\text{KD}+\text{SDM}}{2}. \end{array}$$

### 2.4. Gaussian Interaction Spectrum Nuclear Similarity for Microbes

In the same way, the Gaussian interaction similarity *m*_*i*_ and *m*_*j*_ between microorganisms can be obtained as the Gaussian kernel similarity matrix (KM) between microorganisms.

(7) $$\begin{array}{c} \text{KM}\left(m_{i},m_{j}\right)=\exp\left(-\gamma_{\text{m}}{\left|\left|\text{VP}\left(m_{i}\right)-\text{VP}\left(m_{j}\right)\right|\right|}^{2}\right).\\ \gamma_{m}=\frac{\gamma_{m}^{\prime }}{1/nm\sum_{i=1}^{nm}{\left\|\text{VP}\left(m_{i}\right)\right\|}^{2}}. \end{array}$$

where *γ*_*m*_′ is usually set to 1.

### 2.5. Building a Heterogeneous Network

A heterogeneous network can be expressed as *G* = (*D*, *E*), where *D* represents 331 of all diseases and microorganisms and *E* represents the interaction of microorganisms and microorganisms, diseases and diseases, and diseases and microorganisms. The heterogeneous network is represented by *n*∗*n* adjacency matrix *A*, where *n* represents the number of diseases and microorganisms. By the similarity between the microorganisms (KM) and the similarity between the diseases (KD), the coefficients of similarity can construct a heterogeneity network. Then, for each adjacency matrix *A*, if there is an interaction between *A*_*i*_ and *A*_*j*_, the *i*-th row and *j*-th column are set to 1, otherwise set to zero. Normalize adjacency matrix *A*:

(8) $$\begin{array}{c} A_{\left[i,j\right]}^{\prime }=\frac{A_{\left[i,j\right]}}{\sum_{k=1}^{n}A_{\left[k,j\right]}}. \end{array}$$

### 2.6. Restart Random Walk Algorithm in Both Directions

Through heterogeneous networks, random walks are used to find potential genetic association data between diseases or microorganisms. By randomly walking to convergence, you can get the probability of a disease or microbe at every point in the heterogeneous network. The relationship between microorganisms and diseases is indicated by calculating the correlation between the probability distributions of disease and microorganisms.

For a disease, we list all relevant diseases and microorganisms in our known data set, and then our related diseases and microbial collections are the seeds of the disease. Among them,

(9) $$\begin{array}{c} P_{\text{dis}}={\left[\psi_{\text{dis}¯1},\psi_{\text{dis}¯2},\cdots ,\psi_{\text{dis}¯n}\right]}^{T}. \end{array}$$

Among them, the disease-related diseases and microbial aggregates *ψ*_dis¯*i*_ were set to 1, and the others were set to zero. Normalize *P*_dis_:

(10) $$\begin{array}{c} P\prime_{\text{dis}\left[k\right]}=\frac{P_{\text{dis}\left[k\right]}}{\sum_{k=1}^{n}P_{\text{dis}\left[k\right]}}. \end{array}$$

Similarly, we list all relevant diseases and microorganisms for a certain microbe, we know the data set, and then, we related diseases and microbial collections as *P*_mic_.

Begin random walks and randomly access adjacent genes in each time scale (*t*⟶*t* + 1). State probability *P*_*t*+1_ at time *t* + 1:

(11) $$\begin{array}{c} P_{t+1}=\left(1-r\right)A^{\prime }P_{t}+rP_{0}, \end{array}$$

where *P*_*t*_ is the probability of time *t* and *r* is the probability of restart. According to previous studies, we set *r* to 0.7 [19]. If the difference between *P*_*t*_ and *P*_*t*+1_ is less than 10^−6^ used in the previous study, the process will reach a steady state [20, 21]. By using the mapped set *P*_dis_ as the seed of the disease and the mapped set *P*_mic_ as the seed of the microbe, we implemented a two-way random walk algorithm to obtain the association probability score_*d*_ with disease as the random seed and the association probability score_*m*_ with microorganism as the random seed. The association probability score between the disease *d*_*i*_ and the microorganism *m*_*i*_ is finally obtained by linearly combining the two predicted probabilities.

(12) $$\begin{array}{c} \text{Score}={\beta \text{score}}_{m}+\left(1-\beta \right){\text{score}}_{d}, \end{array}$$

where *β* represents the parameter of the linear combination; we set the default value to 0.7.

## 3. Results

### 3.1. Performance Evaluation

To verify the predictive performance of DRWHMDA, we implemented 5-fold CV and global LOOCV on the model based on the HMDAD database. In each 5-fold CV, the known correlation matrix *Y* is divided into 5-folds; then each fold is taken as a test set, and the remaining 4 folds are treated as a training set. On the other hand, in the global LOOCV, each known microbial-disease association is sequentially excluded from the test, and other microbial-disease associations are used as training samples for model learning. Specifically, all microbial-disease pairs without known evidence of correlation will be considered candidate samples. Further obtain the rank of each missing test sample relative to the candidate sample. Test samples with a prediction level above a given threshold will be considered to have successfully predicted. We evaluated the predictive performance of the model based on the AUC value of the area under the curve of the receiver. Specifically, only test samples ranked above a certain threshold can be considered correct predictions. We then set the true-positive rate (TPR, sensitivity) and false-positive rate (FPR, 1 − specificity) as the horizontal axis and the vertical axis, respectively. Therefore, we can draw a receiver operating characteristic (ROC) curve composed of points corresponding to different thresholds and then obtain the area (AUC) under the ROC curve. A model with an AUC value equal to 0.5 is equivalent to random prediction. When the AUC takes a maximum of 1, the model has excellent prediction performance. In other words, when the value of AUC is greater than 0.5 and less than 1, the larger the value is, the better the prediction performance of the model.

As shown in Figure 2, the 5-fold CV value of DRWHMDA was 0.8676, which was significantly larger than those of KATZHMDA (0.8382), LRLSHMDA (0.8493), and ABHMDA (0.8571). What was more, the global LOOCV value of our model reached 0.8897, which was also obviously better than those of KATZHMDA (0.8644), LRLSHMDA (0.8843), and ABHMDA (0.8861). These results confirmed the superior prediction performance of DRWHMDA.

To investigate the selection of restart probability *r* for the performance of DRWHMDA, we set various values of *r* ranging from 0.1 to 0.9 and calculated AUC in the framework of 5-fold CV. As shown in Table 1, as the restart probability r gradually increases, the prediction performance obtained through DRWHMDA increases first and then decreases.

### 3.2. Case Study

In the present study, double-ended random walks were used to screen candidate microorganisms for all the investigated diseases. To further evaluate the predictive performance of DRWHMDA, we included 10,038 unknown samples in HMDAD, involving 39 diseases and 292 microorganisms. The corresponding unknown samples are classified and ranked by the DRWHMDA algorithm, and it is verified whether the relevant literature has verified the association between the top ten microorganisms and the disease under study. Among them, an independent case analysis was performed on colon cancer and asthma.

### 3.3. Relationship between Colon Cancer and Microorganisms

According to previous research, the intestinal microflora is the most complex, and it is most closely related to various behavioral diseases in humans. Imbalance of the human intestinal microbial flora can lead to autoimmune diseases [22], obesity [23, 24], inflammatory bowel disease (IBD) [25], diabetes [26], and even cancer [27, 28]. According to the world's leading cancer statistics report, colon cancer has been a high-risk area for men and women over the past few decades [29]. Therefore, it is necessary to study the pathogenesis of colon cancer in order to explore new treatment methods. More and more evidences show that the imbalance of microbial community is closely related to the occurrence and development of colon cancer. For example, in the sequence analysis of 16S rRNA gene V3 region in patients with sporadic colorectal cancer, the protein bacteria are insufficient [30]; Staphylococcus produces tannase; its activity may be related to the development of colon cancer [31]. Compared with noncancerous tissues, Lactococcus and Fusarium are more abundant in cancerous tissues, and Pseudomonas and Escherichia coli are less abundant [32]. We applied DRWHMDA to the first case study of colon cancer. Of the top 10 predicted microorganisms, 9 have been validated based on recent experimental literature (see Table 2). Evidence suggests that Clostridium difficile- (first in the prediction list) associated colitis is a known complication of colon and rectal surgery and can increase morbidity and mortality during surgery, thereby increasing hospital stay time and costs [33].

### 3.4. The Relationship between Asthma and Microbes

Asthma is a common chronic inflammatory disease of the lungs and is generally thought to be caused by a combination of genetic and environmental factors. According to the latest statistics, the incidence of asthma has been rising in recent decades, with the number of asthma patients increasing from 183 million in 1990 to 242 million in 2013. Infection by pathogenic microorganisms (especially viruses, chlamydia, mycoplasma, and mold) is one of the main causes of severe asthma [34–37]. For example, studies have shown that Proteus accounts for a higher proportion of microorganisms in asthma patients and that Firmicutes are reduced in asthma patients compared to normal people. Moreover, there is evidence that when the hypopharyngeal area of a newborn is infected with Streptococcus pneumoniae, the risk of developing asthma is increased compared to uninfected [38, 39]. Therefore, research on asthma-related microorganisms is crucial and will help us to gain a deeper understanding of the pathogenesis and treatment of asthma. Prioritizing candidate microorganisms by implementing DRWHMDA, recent clinical evidence successfully validated 9 of the top 10 predicted microorganisms (see Table 3). As for the top five confirmed asthma-associated microorganisms, Clostridium difficile and Staphylococcus aureus (No. 1 and No. 5 in the prediction table) were found to be increased in number in airway concentrations in asthma patients, while Firmicutes and Actinomycetes were found to be reduced [40]. Importantly, the XIVa subclass of Clostridium globosum (No. 3 in the prediction table) has been proven to be an early indicator of future asthma, help prevent and diagnose asthma, and provide guidance for clinical treatment.

For clarity, we illustrate in Figure 3 the association network of the top 10 predicted microbial candidates for two diseases. It is worth noting that some top candidates were found to be related to several diseases. For example, both Fermicket and Clostridium have been documented to prove that they are related to the occurrence of asthma and colon cancer at the same time.

## 4. Discussion

Over the years, a lot of evidence has shown that microorganisms living in the human body are closely related to human life activities and human diseases. Abnormal levels of specific microorganisms are closely related to the development of various human diseases. Microbial disease-related knowledge can provide valuable insights into understanding complex disease mechanisms and preventing, diagnosing, and treating various diseases. However, little work has been done to predict microbial candidates for large-scale human complex diseases. Therefore, in this paper, a computational model based on known microbial-disease correlation is proposed. A microbial similarity network and a disease similarity network are constructed using Gaussian kernel similarity. Using the existing experimentally validated associations, we connected the two networks. The double-ended restart random walk method is used to walk on the network, and the correlation probability order representing the candidate microorganism-disease association is obtained. The construction network with different correlations is applied to the optimization of prediction performance, and the optimal prediction parameters are obtained. The results show that DRWHMDA achieved average AUC reliability performance of 0.8676 and 0.8897 in the 5-fold cross-validation and LOOCV framework, respectively. Given its good predictive performance, we believe that the model can be used as one of the effective tools to accelerate biomedical identification of underlying disease-related microorganisms.

Although DRWHMDA has achieved satisfactory results, this method still has some limitations. First, we only use Gaussian kernel similarity to construct a similarity network which is too simplistic. Improving the predictive performance of DRWHMDA by integrating disease or microbe similarity from multiple data sources (such as sequence similarity) may help. Secondly, as more and more microbes and disease associations are identified, collecting more validated data will help us conduct further research. Finally, we experimentally verify candidate microbes related to the disease, and some have not been verified in the literature, because the verification of these candidate microbes through biological wet experiments will also be one of the important directions for our subsequent research.

## 5. Conclusion

The main goal of the current research is to predict the microorganisms that may be related to the disease through the calculation method, thereby reducing the verification cost of the biological wet experiment, so that people can more deeply explore the impact of microorganisms on human complex diseases. Therefore, this paper proposes a calculation model of microbial disease correlation based on double-ended random walk. The results show that DRWHMDA has achieved more reliable and stable prediction performance than other algorithms. We believe that the model can be used as one of the effective tools for accelerating biomedical identification of potential disease-related microorganisms.

## Figures and Tables

**Figure 1:** The workflow of DRWHMDA for inferring potential microbe-disease associations.

**Figure 2:** The ROC curves for DRWHMDA and other approaches in microbe-disease association prediction for 5-fold cross-validation and global LOOCV.

**Figure 3:** The network of the top 10 predicted associations for the two diseases via DRWHMDA. The dotted line indicates that it has not been confirmed by the literature.

**Table 1:** Prediction AUCs of DRWHMDA at different choices of restart probability *r*.

DRWHMDA	AUC	DRWHMDA	AUC
*r* = 0.1	0.8511	*r* = 0.6	0.8684
*r* = 0.2	0.8513	*r* = 0.7	0.8674
*r* = 0.3	0.8525	*r* = 0.8	0.8666
*r* = 0.4	0.8597	*r* = 0.9	0.8590
*r* = 0.5	0.8695		

**Table 2:** The 10 microbes predicted to be most likely to be associated with colon cancer.

Microbe	Evidence
*Clostridium difficile*	PMID:21152135
*Helicobacter pylori*	PMID:22294430
*Protein bacteria*	PMID:25699023
*Prevotella*	PMID:25699024
*Staphylococcus aureus*	Unconfirmed
*Clostridium globosum*	PMID:18237311
*Fermicket*	PMID:25699024
*Bacteroides*	PMID:25699024
*Actinomycetes*	PMID:26811603
*Clostridium*	PMID:19807912

**Table 3:** The 10 microbes predicted to be most likely to be associated with asthma.

Microbe	Evidence
*Clostridium difficile*	PMID:25974301
*Fermicket*	PMID:23265859
*Clostridium globosum*	PMID:21477358
*Actinomycetes*	PMID:23265859
*Staphylococcus aureus*	PMID:12743582
*Lactobacillus*	PMID:20592920
*Clostridium*	PMID:21477358
*Burkholder*	PMID:24451910
*Gracilariaceae*	PMID:17433177
*Lachnospiraceae*	PMID: 27433177

## Data Availability

The database used in this study was downloaded from the Human Microbe-Disease Association Database (HMDAD, http://www.cuilab.cn/hmdad).
